The article "Correlation of HMGB1, PON-1, MCP-1, and Periodontal P. gingivalis with Amniotic Fluid Fecal Dye" was published in 2022. Journal: J Healthc Eng.

# Correlation of HMGB1, PON-1, MCP-1, and Periodontal *P. gingivalis* with Amniotic Fluid Fecal Dye

**DOI:** 10.1155/2022/3143102

**Published:** 2022-02-22

**Authors:** Zhen-Ai Jin, Ying Li, Wei-Bing Chen, Yu-Ying Wang, Yi-Kun Zhao, Xiang-Lan Sun, Jia-Jun He, Guo Jie, Yu-Mei Sun

**Affiliations:** ^1^Department of Pediatrics, Affiliated Hospital of Yanbian University, 1327 Bureau Street, Jilin, Yanji, China; ^2^Neonatology Department, Rizhao People's Hospital of Jining Medical University, No. 126,Taian Road, Rizhao, Shandong, China; ^3^Jilin Provincial People's Hospital, 1183 Gongnong Street, Chaoyang, Changchun, China; ^4^Obstetrical Department, Rizhao People's Hospital of Jining Medical University, No. 126,Taian Road, Rizhao, Shandong, China; ^5^Department of Obstetrics, Affiliated Hospital of Yanbian University, 1327 Bureau Street, Yanji, Jilin, China; ^6^Department of Neonatology, Dalian Women and Children's Medical Center (Group), No. 1 Dunhuang Road, Dalian Liaoning, China

## Abstract

**Background:**

This paper aims to investigate the correlation between high mobility group protein-1 (HMG-b1), antioxidant enzyme-1 (paraoxon-1, PON-1), monocyte chemoattractant protein-1 (monocyte chemoattractant protein-1, MCP-1), *P. gingivalis*, and MSAF.

**Materials and Methods:**

The total sample size comprised of 73 cases in both groups. These patients were further subdivided into 2 groups: the MSAF group and the control group. 38 women were in the MSAF group and 35 women with term amniotic fluid serum were in the control group. The MSAF group was selected as a full-term singleton amniotic fluid fecal infection group. Clinical data were collected, and specimens were collected. Fecal staining of amniotic fluid and full-term amniotic fluid removes the placenta and umbilical cord blood. The expression of HMGB1 in the placenta was observed by immune-histochemical staining of MSAF and control groups. The content of PON-1 in cord blood was determined by ELISA.

**Results:**

Correlation between maternal and neonatal clinical data and MSAF was done; MSAF group mean gestational age was 41.38 ± 1.40 weeks; control group mean gestational age was 39.20 ± 1.24 weeks. This study found no correlation between the birth weight, maternal age, sex, first/transmaternal, hyperthyroidism, hypothyroidism, and anemia between the MSAF and control group with nonsignificant *P* value (*P* > 0.05). However, the fatal age, gestational diabetes, gestational hypertension, umbilical cord abnormalities, placental abnormalities, and neonatal asphyxia factors were statistically different with a significant *P* value of <0.05 between both groups. HMGB1 and Periodontal *P. gingivalis* are mostly expressed in placental trophoblast, vascular endothelial cells, and amniotic epithelial and interstitial cells. After HE staining of 72 placentas by HE in MSAF and control, 6 had acute chorioamnionitis (5.1 control), 32 had chronic (23.9), 35 had abnormal placentas, and three in MSAF had chorionic columnar metaplasia. In immune-histochemistry experiments, the HMGB1 expression intensity of placental tissue was higher in the MSAF group (*P* < 0.05); however, the level of PON-1 was lower in the MSAF group as compared to the controls (*P* < 0.05).

**Conclusions:**

Gestational age and placental abnormalities are clinical high-risk factors for MSAF. HMGB1, PON-1, MCP-1, and Periodontal *P. gingivalis* may be involved in the development of MSAF, suggesting an oxidative/antioxidant imbalance with inflammation, and may be one of the mechanisms for MSAF development.

## 1. Introduction

In recent years, the birth rate of high-risk pregnant women and critical newborns has been increasing, and the perinatal period of pregnant women has become the focus of attention. Clinically, the MSAF is defined as follows: when stimulated by a variety of causes, it makes fetal intestinal peristalsis, anal sphincter tension decreases, fetal meconium with intestinal peristalsis into the amniotic fluid, originally bright, and translucent amniotic fluid presents different degrees of turbidity, thick, and with the degree of difference, color can appear light green to dark brown change [1, 2]. The theory of the cause and mechanism of MSAF is not unified. At present, there are theories of fetal maturity and umbilical cord extrusion at birth, as well as the theory of fetal intrauterine distress put forward by many scholars. Meconium-stained amniotic fluid (MSAF) occurs when there is a passage of the fetal colonic contents into the amniotic cavity. The frequency of this condition increases as a function of gestational age. The frequency of MSAF ranges from 5% to 20% [3].

The presence of meconium predisposes to meconium aspiration syndrome (MAS) which only occurs in 5% of all neonates born to mothers with MSAF. MSAF is a risk factor for clinical chorioamnionitis, neonatal hypoxic-ischemic encephalopathy, neonatal sepsis, seizures, and cerebral palsy. Therefore, the presence of MSAF is considered a warning sign by obstetricians, even though most neonates do not have evidence of hypoxia or metabolic academia [4]. MSAF can lead to complications such as intrauterine hypoxia and neonatal asphyxia; due to continuous hypoxia of irreversible damage to brain nerves and other organs, such as meconium inhalation syndrome (meconium aspiration syndrome, MAS), hypoxia and ischemic encephalopathy, etc., can be life-threatening when severe [4]. Wu Meiyan's [5] study pointed out that the amniotic fluid fecal infection is more prone to meconium inhalation syndrome, which further revealed that it is more prone to poor prognosis in newborns. At present, few related studies of MSAF and intrauterine inflammation have been reported. The etiology and pathogenesis of MSAF have not been clarified, and increasing attention has been paid to the search for MSAF markers. Through studies of the placenta and umbilical cord blood-related problems, the correlation between intrauterine inflammation and amniotic fluid fecal infection is of certain research value and significance.

Studies have pointed out that [6] MSAF patients had a chorionic amnionitis (chorioamnionitis, CA) probability of more than 50% associated with intrauterine infection. CA is one of the risk factors of intrauterine infection, and microbes entering the amniotic cavity may cause MSAF, while inflammation of the placenta may cause MSAF. Placental lesions can be classified into acute and chronic placental lesions. Acute lesions are mostly related to infection, and chronic placental lesions could be caused by bacteria, viruses, environmental pollution, and other related factors. In Chen Lifen et al. [7], the length of MSAF was found to be extremely closely related to placental lesions. Some researchers believe that intrauterine inflammation is not related to MSAF, so there is some controversy. In clinical work, intrauterine inflammation can be attributed to placental inflammation, umbilical cord inflammation, and fetal membrane inflammation. Studying its interlocality with MSAF can further investigate the occurrence mechanism of MSAF development.

HMGB1, PON-1, MCP-1, and Periodontal *P. gingivalis* are inflammatory factors studied associated with MSAF. All these factors have been involved in the occurrence of inflammation, related to oxidative damage mechanism; however, very less studies and reports are conducted in this regard.

HMGB1, one member of the Alertin family, induces the occurrence of an inflammatory response or the repair of stress trauma to initiate host defense. Relevant studies have found that the generation and release of cytokines can change the signaling regulation inside and outside the cell, thus leading to the occurrence of inflammation and the repair after stimulation [8]. Qiu Xiaoyuan [9] believed that increased levels of HMGB1 expression can aggravate the inflammatory response in the placenta. When the body encounters an infection, HMGB1 can be secreted by immune cells. The signaling pathway is initiated by triggering an inflammatory response by binding to the Toll-like receptor 4 (Toll-like receptor 4, TLR4), as well as to the late glycosylation end-product receptor (Receptor for advanced glycation end products, RAGE).

PON-1 is a member of the antioxidant enzyme family with anti-inflammatory effects, associated with antioxidative stress and with the pathogenesis of numerous diseases. The amount of PON-1 at the site of expression is reduced, causing an oxidative stress response, leading to the occurrence of inflammation [10].

MCP-1 is a chemokine with chemotactic monocytes, macrophages, and T lymphocytes, involved in the inflammatory response, associated with apoptosis, the occurrence and progression of pregnancy diseases, and premature fetal membrane rupture.

Periodontitis in pregnancy should not be confused with pregnancy gingivitis. Pregnancy gingivitis is a common, reversible condition of gingival inflammation associated with high levels of estrogen and blooms of microbial species such as *P. gingivalis*. In periodontitis, the modification of the microbial composition is unrelated to pregnancy status or pregnancy hormones. When good oral hygiene practices are implemented, pregnancy gingivitis resolves within a few months of birth with no permanent changes in CAL. The presence of microbial invasion of the amniotic cavity by *P. gingivalis* could indicate a role for periodontal pathogenic bacteria in pregnant women with a diagnosis of threatened premature labor.

In this study, clinical risk factors of MSAF were analyzed by maternal and neonatal clinical data. The basic aim of the study was to explore the correlation of HMGB1, PON-1, MCP-1, and *P. gingivalis* with MSAF.

## 2. Materials and Methods

### 2.1. Collection of Clinical Data Specimens and Data

Clinical case data of amniotic fluid fecal-stained newborn and normal newborns born were collected from the Affiliated Hospital of Yanbian University.

Placenta and cord blood from the term women with an MSAF collection were set as MSAF groups, while women with term amniotic fluid collection were treated as control groups. Placental pathology was examined by HE staining, HMGB1 expression levels in placental tissue were measured by immunohistochemistry, PON-1 content in cord blood was measured by ELISA, and MCP-1 content in cord blood was determined by flow cytometry.

Specimen collection has been discussed by the Ethics Committee of Affiliated Hospital, Yanbian University to collect placenta and cord blood stained with term amniotic fluid stool delivered from January 2018 to December 2019. The total sample size was comprised of 73 subjects, 38 women in the MSAF group, and 35 women with term amniotic fluid serum in the control group. After specimen collection, all the placentae were stained with HE.

Placental collection method and storage: after the delivery of the maternal placenta, the placenta was extracted and fetal membrane tissue of about 3 cm× 4cm was collected. A 4% formaldehyde solution was taken for sealing and fixation. Paraffin and wax blocks were sectioned, 4 pieces with each cut thickness of 4–6 *μ*m, then sealed, and dried.

Process of umbilical cord blood collection: after delivery of the newborn, before breaking the umbilical cord from the mother, the umbilical cord was cut, and 5 ml of the blood from the lateral umbilical vein was collected with a procoagulation tube. After centrifugation and centrifugation, the upper serum was collected, recorded with specimen information and numbers, and stored in the-80 °C refrigerator.

### 2.2. Degree of MSAF and Diagnostic Criteria of CAM

#### 2.2.1. The Standard of MSAF

Clinically, the amniotic fluid dung dye can be divided into 3°, from light to heavy and further, I degree, II degree, and III degree. I degree: light green, thin quality, and no faecium residue. Degree II : dark green, yellow-green, and relatively thick quality. Degree III : brown, dark yellow, thick, small amount, and visible granular meconium [11]. All the MSAF groups were stained with measured feces in this experiment.

#### 2.2.2. The Diagnostic Criteria for CA

CA is further divided into acute and chronic chorioamnionitis. Acute chorioamnionitis could have neutrophils in the villus connective tissue, amniotic membrane, or chorionic plates. In chronic chorioamnionitis, lymphocytes infiltrate in the chorionic trophoblast and chorionic amniotic connective tissue [12].

#### 2.2.3. Main Instrument, Equipment, and Reagents

The main instrument, equipment, and reagents used in the study have been mentioned in Table 1.

#### 2.2.4. Reagent

*Cell Analysis Kit.* High-throughput liquid-phase protein quantification reagent of human CXCL8/IL-8, CCL5/RANTESCXCL9/MIQ, CCL2/MCP-1, CXCL10/IP-1 cells: Becton, Dickinson, and Company.

Epidemiological histochemical experimental reagents:

1. Rabbit anti-human HMGB1 clonal antibody: Cell Signaling Technology reagent agent
2. DAB Kit: Abcam Reagent, Inc.
3. PV9000 Kit: Abcam Kit Company, containing reagent 1: endogenous peroxidase blocker; reagent 2: reaction enhancer; Kit 3: HRP-enhanced goat anti-mouse/rabbit IgG polymer

*ELISA Experimental Reagent.* PON1 Quantitative ELISA Kit : Shanghai Enzyme Union Biotechnology Co., Ltd. The ELISA experimental reagents have been depicted in Table 2.

### 2.3. Experimental Methods

#### 2.3.1. Detection Steps of the Flow Cell Assay

1. Clean the flow cytometry to ensure the normal function of each instrument detection channel.
2. Prepare standard solution and dilution: take 4 ml standard dilution and freeze ophil dried to mix with the test tube, which is the original liquid, and rest for 10 min. Nine standard tubes were set and one was blank, and the standards were subjected to proportional fold dilutions and added to 10 tubes and labeled S1–S 10. First take 300 ul from the raw liquid into the S1 tube, mix; then move from the S1 tube to 300 ul, and so on, until you move to the S10 tube. The dilution ratio and corresponding concentrations are shown in Table 3.
3. Prepare capture microsphere suspension: IP-10 microsphere suspension was added for 1010 ul to MCB tube, the supernatant was centrifuged for 5 min, and serum was collected. Resuspension and incubation were done in light at room temperature for 20 min.
4. Take serum which has to be measured and further added to the tube for the test; microsphere suspension was added to standard products and serum samples to be measured and incubated for 3h at room temperature
5. Washing: add washing buffer for 1 ml to each tube, and the supernatant was discarded. A 300 ul resuspension microball was added to each tube.
6. The final standards and samples are analyzed for statistical data.

#### 2.3.2. ELISA Method

1. Sample serum: -80 °C, dissolved at room temperature, with shaking.
2. Standard product and number: take standard product reagent, prepare 10 standard holes, and mark S1–S10. The same concentration was added to each two adjacent pore droplets such as S1, S2, and 50 *μ*l, with concentrations of 120, 80, 40, 20, and 10 nmol/mL, respectively.
3. Set blank holes and additional samples: set as B1 and B2, except for blank holes; add 50 *μ*l sample to each sample hole to be tested.
4. HRP: add 50 *μ*l of labeling reagent to each well.
5. Incubation: after gently shaking, the plate membrane was sealed and incubated in a 37°C incubator for 1 hour.
6. Flushing: get rid of the liquid in the hole, fill with washing liquid, repeatedly wash and pat dry, and repeat 5 times in this way.
7. Color display with the color developer: add color developer A, B50 *μ*l, 37°C incubators in each well to avoid light for 10 minutes.
8. Color termination: gently for 50 *μ*l, in each well.
9. OD value of each well by computer.

### 2.4. The HMGB1 Immunohistochemical Staining Results Were Determined

HE staining mainly observed the morphology and pathological changes of the placenta and fetal membrane. In the placenta, HMGB1 is mainly localized in placental trophoblast, vascular endothelial cells as well as amniotic epithelial and stromal cells. The nucleus is positive in blue, and the cytoplasm is brown; negative if the nucleus, cytoplasm, or membrane is shown in blue[13]. Color intensity: The positive intensity of positive cells in each slice was 0 colorless, 1 pale yellow, 2 brown, and 3 dark brown. The average of positive cells: the percentage of positive cells was 0, positive cell <25% 1,25%–50% 2,> 50% was 3; the sum of positive cells and color intensity: 0–1; 2–3 (+); 4–5 (++), and 6 (+++).

### 2.5. Statistical Methods

All of the data were analyzed using SPSS 26.0 statistical software. Study data were analyzed using an independent sample *t*-test, grade data were analyzed using the nonparametric test, and *P* < 0.05 was statistically significant. Risk factors analysis was performed using logistic regression analysis.

## 3. Results

### 3.1. Comparison of Clinical Data between the MSAF and Control Groups

The total sample size comprised of 73 subjects. In the MSAF group, there were a total of 38 subjects, 22 men, 16 females, with the mean gestational age being 41.38 ± 1.40 weeks, and the control group was comprised of a total of 33 subjects, 19 men, 16 females, with the mean gestational age being 39.20 ± 1.24 weeks. The gender, birth weight, maternal age, initial/transmaternal, and gestational history were nonsignificant between both the groups (*P* > 0.05). However, gestational age, gestational diabetes, gestational hypertension, umbilical cord abnormalities, placental abnormalities, and neonatal asphyxia were significant between the groups (*P* < 0.05), shown in Table 4.

Logistic regression analysis of the risk factor analysis in the MSAF group and gestational age and placental abnormalities were high-risk factors for amniotic fluid fecal staining, with OR being 2.639 (95%CI:1.646–4.231) and 4.506 (95%CI:1.034–19.631), respectively, and positively related (Table 5).

### 3.2. Comparison of HMGB1 Expression and PON1, MCP-1, and *P. gingivalis* Content between the MSAF Group and the Controls

#### 3.2.1. HMGB1 Expression in the Placental Tissues of Both the MSAF and Control Groups

HMGB1 is mostly expressed in placental trophoblast, vascular endothelial cells, and amniotic epithelial and interstitial cells. The expression intensity of HMGB1 in the MSAF group was higher than in control tissues and was statistically significant (*P* < 0.05) as shown in Figures 1 and 2 and Table 6.

#### 3.2.2. Comparison of Umbilical Cord Blood PON1 Content in the MSAF and Control Groups

Cord blood PON1 content in the MSAF group was 80.40 ± 24.67 nmol/mL and in the control group was statistically significant (*P* < 0.001) as shown in Table 7.

#### 3.2.3. Comparison of MCP-1 Plots and Content of Cord Blood in MSAF and Control Groups

Cord blood MCP-1 content was 271.10 (174.35–326.62) pg/mL, and the control was 104.89 (50.15–184.19) pg/mL, which was statistically significant (*P* < 0.001), shown in Figures 3 and 4 and Table 8.

### 3.3. Results of Placental HE Staining in Both the MSAF and Control Groups

After HE staining of 72 placentas, six had acute chorionic amnionitis (5 in MSAF, 1 in control), 32 had chronic chorioamnionitis (23 in MSAF, 9 in controls), 5 had nonabnormal placentas, and three in MSAF had chorionic amniotic columnar metaplasia (Figures 5-8).

## 4. Discussion

MSAF refers to the fact that when the fetal fetus is stimulated differently in utero, the intrauterine fetal intestinal peristalsis is enhanced, and when the anal sphincter is relaxed and the meconium is discharged into the amniotic fluid, this makes the amniotic fluid brown and yellow-green and then becomes cloudy and thick [14]. Fetal hypoxia causes intestinal peristalsis, the relaxation of the anal sphincter, and the release of meconium in the amniotic fluid. Meconium can also be sucked out in the first breath at birth, with studies suggesting that meconium induced direct alveolar damage through inflammatory responses and damaged lung parenchyma and endothelial cells and that 3% to 12% of infants born with MSAF would develop MAS, characterized by characteristic X-ray plaque shadows and respiratory distress and often exacerbated by pulmonary hypertension [15]. By collecting clinical data from pregnant mothers and newborns, this study found no difference between gender, birth weight, maternal age, maternal age, and maternal and gestational history, but gestational age, gestational diabetes, gestational hypertension, umbilical cord abnormalities, placental abnormalities, and neonatal asphyxia were statically significant. The gestational age and placental abnormalities were risk factors in the MSAF group and showed a positive correlation, indicating that the greater the gestational age, the more likely to develop MSAF. Lu Shaoxia et al.'s [1] study pointed out that simple amniotic fluid dung infection may not cause fetal distress. In 276 pregnant women with MSAF, the gestational week was found to be a high-risk factor for MSAF, with the incidence of pregnant women over 40 weeks, significantly greater than 38 weeks. Wang Li et al.'s [16] study showed that pregnant mothers had a higher incidence of gestational diabetes and preeclampsia in the MSAF group than in the normal group. MSAF can cause intrauterine oxygen and chronic hypoxia in the newborn and can cause different damage to the respiratory, circulation, and digestive systems of the nervous system of the newborn [17]. The above views are consistent with the present study. In the current study, umbilical cord abnormalities may also be the influencing factor of MSAF, spiral umbilical cord and knot, and tight winding, the umbilical cord is too short, and the incidence of placental inflammation and MSAF is significantly increased [17, 18]. MSAF can be classified into primary and secondary contamination. After the fetal membrane rupture, amniotic fluid is feces, which is primary. After the fetal membrane rupture, the amniotic fluid is clear; along with the progress of the production process, the amniotic fluid gradually changes from brightening to feces dye, for secondary pollution [19]. Secondary meconium contamination cord was associated with meconium neonatal fetal distress and other poor neonatal prognoses, and primary amniotic fluid meconium contamination was associated with adverse outcomes [20]. Severe cases can die early in the newborn [21]. Microbial invasion of the amniotic cavity in placental inflammation increases the incidence of MSAF [22]. At present, the mechanism of amniotic fluid dung dyeing is unclear, and studying the correlation of inflammatory factors and MSAF can further explore the mechanism of MSAF occurrence.

The main diagnosis basis for diagnosing intrauterine infection is that the pathological testing of CA and the placenta can more effectively detect and judge intrauterine infection [23, 24]. There was chronic inflammation of the placenta, compound trophoblast hyperplasia, and villus interstitial fibrosis in this experiment. There were CA, villus interstitial edema, fibrosis, and compound trophoblast hyperplasia; some studies pointed out that inflammatory cells with long span groups were mainly lymphocytes; that is, chronic inflammation is lymphocytes, and groups with short time span were neutrophils; namely, acute inflammation was mainly neutrophils [25]. In this study, it was shown that the MSAF group was more prone to placental inflammation, mainly with chronic inflammation.

HMGB1 is one member of the Alertin family, is divided in various cells, is an evolutionarily conserved DNA binding protein that acts as Alertin, is translocated to the cytoplasm, and is secreted after injury. Extracellularly, it acts as an inflammatory cytokine [26, 27]. In this study, HMGB1 expression in placentas is higher in the MSAF group than in the control by immunohistochemical staining of both placentas. Considering that HMGB1 has been implicated in placental inflammation, high HMGB 1 expression can upregulate the expression of late glycosylation end-product receptor (receptor for advanced glycation end products, RAGE), initiate a positive feedback mechanism, activate NF-*κ*B, to produce a series of inflammatory factors, and exacerbate the inflammatory response in the placenta [28]. HMGB1 may be involved in the occurrence of MSAF. HMGB1 has been associated with pregnancy complications, such as preterm birth and CA [29, 30]. Salihu et al. [31] pointed out that HMGB1 can accelerate partial cellular senescence and enhance contractility in the myometry and expression of inflammatory genes. Endogenous hazard signals activate the Toll-like receptor-2 (TLR-2) and the Toll-like receptor-4 (TLR-4) and play a role in inflammatory diseases. HMGB1 may serve as an endogenous activator of these receptors. HMGB1 promotes neutrophils but not macrophage migration to necrotic tissue. In addition to the active secretion from inflammatory cells, HMGB1 is also passively released from necrotic cells, and HMGB1 from cells at different sites can affect the inflammatory response after necrosis to varying degrees [32]. HMGB1 can promote the release of inflammation, with redox and endogenous cytokines-induced functional extracellular TLR4 mainly expressed in placental compound trophoblasts and fibroblasts. HMGB1 induces macrophages to produce inflammatory cytokines in a redox-dependent manner through TLR4 signaling, affecting cell proliferation, differentiation, and migration [26, 33]. All indicate a correlation with the occurrence of inflammation. HMGB1 can form an immunostimulatory complex. The inflammatory response triggered by HMGB1 may be involved in the placental inflammatory response that can induce the production of transcription factors (e.g., NF-*κ*B) and trigger a local (and subsequently systemic) inflammatory response [34]. TLR2 and TLR4 are associated with MSAF, and in inflammatory cells, the Toll-like receptor (TLR) is combined with its ligand (HMGB1) through the recruitment of linker proteins to strongly activate NF-kB signaling, triggering inflammation [35]. The activity of HMGB1 that depends largely on its redox state, reduces HMGB1 release, and chemically modifies its redox form can improve inflammation as well as tissue damage. A positive correlation was observed between the expression level of reactive oxygen species and the expression of HMGB1 protein [36]. In the MSAF study, HMGB1 expression in the placenta was stronger than in the control group, reliable, and oxidized.

PON-1, a member of the antioxidant enzyme family with anti-inflammatory effects, is an effective antioxidant associated with the pathogenesis of multiple diseases [37]. Multiple pathophysiological diseases are related and also have the damage of degraded organophosphate compounds to the nervous system [38, 39]. Thus, the state of PON1 in vivo can be determined by measuring the levels of enzymatic activity with different substrates [40, 41]. In this study, the PON1 gene is closely related to poison metabolism, and the strength of its activity directly affects the poison metabolism process in vivo. The oxidative stress response is involved in the development of inflammation and is an important cause of the expansion and aggravation of inflammatory response. The interaction of oxidative stress with the inflammatory response is the mechanism of disease development. Oxidative products are produced in normal physiological metabolism, while cells express endogenous antioxidants to remove free radicals and combat the harmful effects of reactive oxygen species products, keeping the oxidation/antioxidant system in a stable, balanced state [42]. PON-1 is a marker in oxidative stress metabolites. In the state of oxidative stress, the measured PON-1 content of cord blood in this study showed lower PON1 activity in the MASF group than normal group, considering the oxidative/antioxidant system imbalance and the occurrence of oxidative stress and inflammation. Shandan et al. [43] pointed out that oxidative stress can cause placenta ischemia and hypoxia and affect the release of inflammatory factors and related enzymes. The possible involvement in the oxidative stress response in causing inflammation may have some relevance to MSAF.

MCP-1 is chemotaxis immune cells that produce corresponding antibodies after stimulation and affect phagocytosis to resist the invasion of foreign microorganisms. In recent years, studies have pointed out labor initiation, preterm birth, and pregnancy-related diseases [44, 45]. Xu Qingyun [46] suggests that elevated MCP-1 in neonatal cord blood may be involved in the development of CA. The main factor of CA is inflammatory factors through signaling; oxidative stress can stimulate inflammation and fetal edema degeneration; edema appeared in this study; there was placental HE staining; three cases had columnar metaplasia and MSAF cord blood MCP-1 higher than the control group and statistically significant difference; for placental HE staining, 3323 cases in the MSAF group had placental CA and mainly chronic chorioamnionitis. Case analysis studies studying preterm birth with MSAF indicated a higher probability of CA compared with the MSAF group [47, 48]. Liu Weiwei [14] pointed out that pregnant women in the MSAF group had a higher probability of neonatal infection than in the CA-free group; CA increased neonatal infection rate, increased intrauterine infection index in the perinatal period, and increased risk of infection during fetal delivery. Yan Lili et al. [49] pointed out that MCP-1 can drive activated macrophages and, with high MCP-1 expression, increases cell adhesion and invasion and aggravates inflammation. In pediatric bronchial asthma, oxidative stress status is correlated with it, among which MCP-1 increases significantly between the onset and remission period in children, pointing out that oxidative stress levels are correlated with the imbalance of inflammatory factors [50]. MCP-1 may have some correlation with MSAF [9].

### 4.1. Limitations

The small sample size is limited, and increasing the sample size can improve the relevant studies.

## 5. Conclusion

The study concluded that gestational age and placental abnormalities are clinical high-risk factors for MSAF. We have found that placental chorioamnionitis may be one of the causes of MSAF. HMGB1, PON-1, MCP-1, and *P. gingivalis* may be involved in the development of MSAF, suggesting an oxidative/antioxidant imbalance with inflammation, and may be one of the mechanisms of MSAF development.

### 5.1. Practical Implications

HMGB1 PON-1, MCP-1, and *P. gingivalis* play an important role in immune responses in MSAF patients [51].

## Figures and Tables

**Figure 1:** Expression of chorionic amniotic HMGB1 (400 ×) in the control group.

**Figure 2:** Expression of chorionic amniotic HMGB1 (400 ×) in the MSAF group.

**Figure 3:** Cord blood MCP-1 content in the control group.

**Figure 4:** Cord blood MCP-1 content in MSAF group.

**Figure 5:** Chorioamnionitis (200 ×).

**Figure 6:** Chorioamnionitis with lymphocyte infiltration (200 ×).

**Figure 7:** Chorioamniotic columnar epithelialization (400 ×).

**Figure 8:** Placental chorioamnionitis edema in the MSAF group (400 ×).

**Table 1:** Instrument name and manufacturer.

	Instrument name	Manufacturer
1	Leica automatic slicer	Leica, Germany
2	PHY-III pathological tissue bleaching oven	Shanghai Changchang Electronics Co., Ltd.
3	Electrothermal constant temperature incubator	Shanghai Yuejin photochemical instrument Factory
4	Digital imaging equipment	Digital imaging equipment
5	Micro oscillator	Xishan Jincheng Instrument Factory
6	Foshan Zhiguang instrument Factory	Foshan Zhiguang Instrument Factory
7	Ultrapure water machine	Shanghai Yuejin photochemical instrument Factory
8	- 80°C refrigerator	Zhongke Meiling company
9	Table type low speed refrigerated multitube centrifuge	Shanghai Anting Scientific Instrument Factory
10	Micropipette	Mettler Toledo Instruments Co., Ltd.
11	BioTek reader	Biotec instruments
12	Incubator	Shanghai Xinmiao Medical Instrument Co., Ltd.
13	Eppendorf micro sampler Eppendorf	Germany
14	Flow cytometry	Beckton, Dickinson

**Table 2:** PON1 quantitative ELISA kit components.

Intracellular kit reagent	
1 Instructions	Sample dilution: 1 bottle (6 ml)
Seal plate film is 2 sheets	Color A and B 1 bottle each (6 ml)
The plate was coated with 96-well plates	Termination solution: 1 bottle (6 ml)
Standard product (concentration of 120, 80, 40, 20, and 10 nmol/mL, respectively) 5 bottles (2 ml)	Concentrate the detergent for 1 bottle (25 ml)
Enzyme labeling reagent 1 bottle (6 ml)	

**Table 3:** List of corresponding concentrations and dilution ratio of standard tubes.

Standard tube number	Corresponding concentration (pg/ml)	Dilution fold ratio
S1 (blank control)	0	0
S2	10	1 : 256
S3	20	1 : 128
S4	40	1 : 64
S5	80	1 : 32
S6	156	1 : 16
S7	312.5	1 : 8
S8	625	1 : 4
S9	1250	1 : 2
S10	2500	1 : 1

**Table 4:** Comparison of birth weight and maternal age of newborns in each group.

Project	MSAF group (n, %)	Control group (n, %)	*χ* ^2^(*t*%)*Z*	*P*
Fetal age (*x* ± *s*)	41.38 ± 1.40	39.20 ± 1.24	7.053	<0.001
Birth weight (*x* ± *s*)	3.55 ± 0.34	3.41 ± 0.40	1.698	0.094
Mother age (*x* ± *s*)	29.50 ± 4.39	30.00 ± 5.11	0.309	0.759
Gender (male/female)	22/16	19/16	1.083	0.298
Early/via maternal	13/25	11/24	0.064	0.804
Pregnancy diabetes	12 (31.6)	4 (11.4)	4.323	0.038
Pregnancy hypertension	15 (39.5)	5 (14.3)	5.811	0.016
Hyperthyroidism, hypothyroidism, and anemia	6 (15.8)	5 (14.3)	0.032	0.858
Abnormal umbilical cord	9 (23.7)	2 (5.7)	4.597	0.032
Abnormal placenta	23 (60.5)	9 (25.7)	8.968	0.003
Neonatal asphyxia	17 (44.7)	8 (22.9)	3.873	0.049
History of fetal protection	9 (23.7)	7 (20.0)	0.145	0.704

**Table 5:** Logistic regression analysis of the risk factor analysis in the MSAF group.

	B	SE	Wald	*P*	OR (95%CI)
Fetal age	0.971	0.241	16.247	<0.001	2.639 (1.646–4.231)
Pregnancy diabetes	1.242	1.371	0.821	0.365	3.461 (0.236–50.808)
Pregnancy hypertension	0.753	1.114	0.457	0.499	2.122 (0.239–18.823)
Abnormal umbilical cord	1.139	1.217	0.876	0.349	3.123 (0.287–33.932)
Abnormal placenta	1.505	0.751	4.020	0.045	4.506 (1.034–19.631)
Neonatal asphyxia	1.295	0.782	2.742	0.098	3.653 (0.788–16.926)
Constant	-40.592	9.827	17.062	<0.001	0.000

**Table 6:** Comparison of HMGB1 expression intensity between the MSAF and control groups.

Group	*N*	HMGB1 expression intensity				*Z*	*P*
		-	+	++	+++		
MSAF group	38	1	7	11	20	6.494	＜0.001
Control group	35	18	15	2	1		

**Table 7:** Comparison of PON-1 content between the MSAF and control groups.

Group	N	PON-1 (nmol/mL)
MSAF group	38	80.40 ± 24.67
Control group	35	95.65 ± 24.33
Z		2.658
*P*		<0.010

**Table 8:** Comparison of MCP-1 content between the MSAF and control groups.

Group	N	MCP-1（pg/mL）
MSAF group	38	271.10（174.35–326.62）
Control group	35	104.89（50.15–184.19）
Z		4.03
P		＜0.001

## Data Availability

The collected data have been included in the study.
